This article has been retracted.

# Analysis of Age and Prevention Strategy on Outcome after Cerebral Venous Thrombosis

**DOI:** 10.1155/2020/6637692

**Published:** 2020-12-14

**Authors:** Xiuli Chu, Jianlin Zhang, Bin Zhang, Yuwu Zhao

**Affiliations:** ^1^Department of Neurology, Shanghai Jiao Tong University Affiliated Sixth People's Hospital, Shanghai, China 200233; ^2^Department of Neurosurgery, Taian Central Hospital, Taian, Shandong Province, China 271000

## Abstract

**Method:**

We identified adult CVST patients in our centers. Functional outcome and prevention strategy were extracted from medical records. Modified Rankin Scale (mRS) ≤ 1 is considered a good functional outcome.

**Results:**

A total of 113 patients were identified. The most common presenting symptoms were headache (86.72%) and nausea/vomiting (56.63%); the top two identified risk factors were local head/neck infection (27.43%) and pregnancy/puerperal period (19.47%). The medical encounter lag time was 0.04 d-120 d. Four enrolled patients were diagnosed as CVST again, and the interval time was 3-8 years from the first time. Thrombus was most frequently seen at superior sagittal sinus (53.10%) and sigmoid sinus (50.44%). 94 (83.19%) of the patients had good outcomes. In the acute phase, 91 (80.53%) patients received low molecular weight heparin, 29 (25.66%) took aspirin, 7 (6.19%) patients were put on low molecular weight heparin and aspirin together. During our follow up (6-24 m), there were 10 (8.85%) patients who suffered from thrombotic event recurrence. For the patients > 40 years old, they tended to suffer from neurological deficit (25.00%) and stupor/coma (16.67%) (*p* > 0.05), with a higher rate of hemorrhage (20.83%) and death (4.16%) when compared with the younger patients (10.77% and 1.53%, separately) (*p* > 0.05).

**Conclusion:**

Functional outcome after CVST appears good. For the patients over 40-year-old, neurological deficit and altered consciousness were more common, accompanied by a higher rate of hemorrhage and mortality. The recurrent rate of CVST was low, longer-term follow up needed. The prevention strategy after CVST was uncertain, further studies needed.

## 1. Introduction

Cerebral venous sinus thrombosis (CVST) is an uncommon cerebrovascular disease. Unlike the arterial stroke, it affects mainly middle-aged individuals and is more common among females [1]. CVST is generally accompanied with a good prognosis, the short-term mortality is <10%, and the majority of patients regain independence in daily living [2, 3]. In the International Study on Cerebral Vein and Dural Sinus Thrombosis (ISCVT) study, the death rate was 8%, 80% of patients recovered well (defined as a score of 0–1 on the modified Rankin Scale (mRS)), and the CVT recurrent rate was 1.5/100 patient per years [4]. Older age (>37 years), male sex, coma, seizure, deep CVST, brain hemorrhage, and concomitant diseases such as hematological pathologies, systemic malignancy, and central nervous system infection were considered to be the risk factors [5]. Antithrombotic medication is the primary acute therapy for CVST, recommended by the American Heart Association and American Stroke Association [6]. However, treatment options remain controversial, and the clinical outcomes are uncertain. Most patients will accompany with a good prognosis, which may affect the patient's compliance with following preventive treatment. Relatively few small studies have investigated long-term outcomes (beyond 1–2 years) and prevention strategies after CVST [7–9].

The aims of this study were to investigate the association between age or prevention strategy with the functional outcome in a double-center patient population. We also explored their risk for recurrent venous thromboembolism (VTE), antithrombotic medication use, and risk for bleeding events.

## 2. Methods

### 2.1. Study Design

This was a double-center retrospective cohort study. Patients were identified from January 2013 to June 2016 at the Shanghai Sixth People's Hospital affiliated to the Shanghai Jiao Tong University and Taian Central Hospital.

The inclusion criteria for this study are (1) CVST is made by clinical diagnosis with magnetic resonance imaging (MRI)/magnetic resonance venography (MRV); (2) age > 18 old years; (3) patient has at least one 6-month follow-up clinical visit after the index event.

We extracted the following information from medical records: demographic information, presenting symptoms (headache, vomiting, papilledema with/without visual loss, other neurological symptoms, or signs), NIHSS score, Glasgow Coma Scale (GCS) score, the imaging information, the location of the thrombus, comorbid medical history, and medication for CVT.

All patients were interviewed at 6 to 24 months by direct interview, or a telephone interview was done if the patient could not show up for an in-person visit. Follow-up data recorded were as follows: headaches, seizures, visual loss, functional outcomes measured by mRS, death, recurrent symptomatic sinus thrombosis (new clinical symptoms with new thrombus shown on MRV), VET or CVST events, pregnancy/abortion during the follow-up period, and antithrombotic treatment.

The primary outcome measures were the mRS. A favorable outcome was defined as mRS 0-1, indicating complete recovery or only mild residual symptoms not affecting everyday life.

### 2.2. Statistical Analysis

Baseline categorical variables will be listed as number (percentage). Baseline normally distributed continuous variables will be reported as mean ± standard deviation (SD), while nonnormally distributed continuous variables will be reported in median (interquartile range [IQR]). Comparisons of continuous variables between the two groups were performed by the two-sample-testify normally distributed with equal variance between groups; otherwise, Wilcoxon rank-sum test would be used. Comparisons of categorical values between the two groups were performed by Chi-square test or Fisher's exact test. A two-sided difference is considered significant if the null hypothesis is rejected at the 0.05 probability level. Statistical analyses were performed using SPSS, version 24.0 (SPSS Inc., Chicago, IL, USA).

## 3. Results

### 3.1. Baseline Patient Information, Presentation

We identified 113 consecutive patients diagnosed as CVST. The median age of patients at diagnosis was 32.50 years (IQR rang 27-48.75): 63 (55.75%) of them were females. The median medical encounter lag time was 5.00 days (IQR range 2.00-10.00). The most prevalent signs and symptoms were headache (86.72%), nausea/vomiting (56.63%), and motor or sensory deficit (22.12%). There were 28 (24.78%) patients who had a NIHHS score > 2. Of the 17 (30.36%) patients, headache was the only symptom they had. For the patients in the cohort, 36 (31.86%) patients were not identified with the specific reasons, 31 (27.43%) patients suffered from central nervous system infection, 22 (19.47%) patients under pregnancy/puerperal period, 14 (12.39%) had coagulation disorder, 8 (7.08%) had systemic prothrombotic disorder, 8 (7.08%) had anemia (all 8 were puerperal patients), 8 (7.08%) patients suffered from hemorrhoids surgery, 3 had malignancy (2.65%), 3 (2.65%) patients had the history of oral contraceptives, 2 (1.77%) had polycythemia, 1 (0.88%) had dural fistula confirmed by digital subtraction angiography (DSA), and 1 (0.88%) patient had dehydration for more than 12 hours (Table 1, Figure 1).

### 3.2. Imaging Findings

For the patients with neuroimaging at admission, combined with the CT/MRV/MRI exam, the results showed that there were 21 (18.58%) patients who showed infarct in CT/MRI, and 17 (15.04%) patients showed hemorrhage. Thrombus was most frequently localized at superior sagittal sinus (53.10%), sigmoid sinus (50.44%), transverse sinuses (48.67%), and straight sinus (7.08%). There were 41.59% patients who had one sinus that clotted, 35.40% patients had two sinuses that clotted, 23.01% patients had more than two sinus involved. Thirty-one patients had the risk factor of local infection, 19 (61.29%) patients localized at superior sagittal, 14 (45.16%) patients localized at transverse sinuses, 14 (45.16%) patients clotted at the sigmoid sinus, and 9 (29.03%) straight sinus. There were 5 (16.13%) patients who had more than two sinuses that clotted, 9 (29.03%) patients had two sinuses that clotted, 17 (54.83%) patients just had one sinus involved (Table 2, Figure 2).

### 3.3. Antithrombotic and Prevention Strategy

In the acute phase, 81 (71.68%) patients received low molecular weight heparin, 15 (25.00%) took aspirin, 10 (8.85%) patients were given warfarin, and 7 (6.19%) patients were put on low molecular weight heparin and aspirin together for combined with other diseases. Within the 113 patients, 5 patients were the recurrence of CVST and in charged into our hospital, the recurrent interval since the first diagnose was 2-8 years, and the recurrent syndrome was headache for all of them. One patient has taken aspirin for prevention, and recurrent 3 years later; two patients did not take medicine, and recurrent 2 and 3 years later, separately; 2 patients had taken warfarin, and recurrent 2 and 8 years later, separately. The median follow-up duration for the entire cohort was 10 (6-24) months. In the following period, 3 patients lost follow-up. By the end of the follow-up, 52 patients (46.02%) had taken warfarin for more than 6 months, 19 (16.81%) patients had taken aspirin instead for more than 6 months, 3 (2.65%) patients had a combination of medication, 8 (7.08%) patients had taken traditional medicine instead, and 28 (24.77%) patients declined to take any specific medication after discharge. Eleven (8.39%) patients experienced thrombotic events recurrently during our follow-up period. Six patients had taken warfarin, 1 patient had taken aspirin, and 4 patients declined to take any medication.

### 3.4. Outcomes

Regardless of treatment strategy, 94 (83.18%) patients achieved a good clinical outcome (mRS 0-1). 4 (3.54%) patients had an intermittent headache, which affected their normal life. 10 pregnant patients all had smooth production. Intracranial hemorrhage (ICH) was the most cited complication, 9 (52.94%) of 17 patients suffered from hemorrhagic events requiring medical attention, which were potentially life-threatening (4 intracranial bleedings, 2 of which were traumatic), although none was fatal (Table 1).

Death was observed in 3 (2.65%) patients: 2 of them died from direct consequences of the indexed CVST in the hospital, the brain edema aggravated by coma, leading to death. 1 patient died from underlying malignancy in the following period.

### 3.5. Subgroup Analysis

Then, we divided the patients according to patients' age (≥40 vs. <40 years old). For the patients over the age of 40, they had shorter medical encounter lag time (median 5.00 days, IQR 2.00-14.00), compared to younger patients (median 4.50 days, IQR 2.25-9.75). They were more likely to suffer from motor or sensory deficit (25.00%) and stupor/coma (16.67%). To identify the risk factors, among the patients over 40-year-old, there were 60.42% of patients who could not find identical reasons (*p* < 0.01). Among the patients under the age of 40, the risk factors were higher in anemia (12.31%, *p* < 0.05), pregnancy/puerperium (33.84%, *p* < 0.05), surgery (12.31%, *p* < 0.05), central nervous system infection (29.23%, *p* > 0.05), and oral contraceptives (4.61%, *p* > 0.05). The patients over 40-year-old were more likely to suffer from hemorrhage (20.83%) and mortality rate (4.16%) compared to younger patients (10.77% and 1.53%, separately), but the results had no significant meanings (*p* > 0.05) (Table 1, Figure 1).

## 4. Discussion

Our study provided data on various aspects of outcomes in a double-center cohort of CVST patients. The recurrence risk for CVST was low. The majority of patients (83.18%) had a favorable outcome (mRS 0-1).

Our results were similar to the results of the ISCVT study (80.0%) [5] and the VENOST study (88.9%) [10], which were the two largest studies of CVST. CVST predominates in children and young and middle-aged adults and rarely happened in elder patients. Some of the risk factors, such as pregnancy, puerperium, and use of oral contraceptives, are no longer present in elderly patients, whereas others such as malignancy and dehydration may be more frequent [5], which may cause the risk factors between each age groups are different and may impact the symptoms and outcome. The ISCVT found that older age (>37 years) was a predictor of poor outcome (mRS > 3) [5]. In our study, we divided the patients according to the age and carried a subgroup analysis. For the patients <40 y, the common risk factors were pregnancy/puerperium, central nervous system infection, anemia, and surgery; whereas for the patients over 40-year-old, there were 60.42% patients who could not find identical reasons, local infection rate were 25.00%, and the coagulation disorder rate reached 12.50%. The ages have influenced the outcome, for the patients ≥ 40 years old had a higher rate of hemorrhage (20.83%) and mortality (4.16%).

Headache is the most common presenting symptom of CVST patients (60%-90%) in many studies [5, 9, 10], and sometimes it may be the sole complaint in a large number of patients [10]. Of the 113 patients, 86.72% experienced headaches, and it was the only symptom in 29 (25.66%) patients. In our study, motor or sensory deficit and altered consciousness were more common in patients aged > 40 years old, whereas younger patients frequently presented with visual field deficit, headache symptoms, and seizure. And the older patients usually ignored the symptoms and unwilling to visit the doctor; unless the symptoms got worse (an unbearable headache), the medical encounter lag time of older patients (median time 5.00 days, IQR 2.00-14.00) was longer than the younger patients (median time 4.50 days, IQR 2.25-9.75). The clinical presentation of our cohort is almost identical to what has been reported in many previous studies.

The most frequently affected sinuses in our cohort were superior sagittal sinus (53.10%), sigmoid sinus (50.44%), and transverse sinuses (48.67%), possibly as a consequence of their morphological inferiority (often being hypoplastic) [11]. These results of the VENOST study showed 73.4% in transverse sinuses, 39.8% in sigmoid sinus, and 38.9% in sagittal sinus [10]. In the ICVST study, the superior sagittal sinus was the most commonly affected (62%), followed by the transverse sinuses (41.2%-44.7%). The association of transverse and sigmoid sinus thrombosis with local inflammation in the nasal, tonsillar, and middle ear area was commonly observed, which was similar to our research; the patients with local infection localized at superior sagittal most. With the increased use of antibiotic treatment, the global incidence of inflammatory phlebothrombosis was reduced, and the outcome became better [12]. In the developing countries, the reported proportion of a local infection in adults with CVST is only 15% [13], and the proportion has decreased to 6% to 12% in the developed world [14], compared with our study (17.86%).

Treatment options remain controversial. The American Heart Association and American Stroke Association have suggested anticoagulation should be started as long as there are no major contraindications, and the patients suggested to continue to receive oral anticoagulation for 3-12 months if the patient exhibits neurological improvement or remain stable [6]. However, until now, we just have limited data to suggest the anticoagulation treatment is safe [9, 15]; there were some studies that come to inconclusive results for the clinical outcome with or without anticoagulation [16, 17]. In the ISCVT study, 83.3% of patients were given anticoagulation drugs, and 5.9% of patients received antiplatelet drugs [5]. In our study, in the acute phase, there were 80.53% of patients who received anticoagulation drugs, and 25.00% of patients received antiplatelet drugs. After the discharge from the hospital, the patients who had taken warfarin decreased to 46.02%, 16.81% patients chose to take aspirin, and 24.77% patients chose to observation without taking any medicine. By the end of follow-up, eleven (8.39%) patients experienced thrombotic events recurrently during our follow-up period. Six patients had taken warfarin, 1 patient had taken aspirin, and 4 patients declined to take any medication. No institutional guidelines are recommended for the use of aspirin, but doctors often prescribe aspirin to patients with no obvious or transient risk factors, or some patients chose to take aspirin for the lower rate of hemorrhage and the complex of regular monitoring of coagulation. Aspirin use may play a role in lowering the incidence of VTE, as aspirin reduces the risk of venous thrombosis by 42% [1, 18]. Further prospective studies are needed, as physicians might have been biased and treated severe clinical presentations more aggressively with anticoagulation, and the patients with other kinds of complications should be considered, for the higher rate of hemorrhage and recurrent rate.

Previous studies showed that the risk of recurrence of a thrombotic event seems to be the highest in the first year after diagnosis [4, 19]. Relatively few small studies have investigated long-term outcome (beyond 1–2 years) after CVST [1, 7]. In our cohort, 5 of the enrolled patients were CVST recurrence, the recurrent interval since the first diagnose was 2-8 years, and the recurrent syndrome was a headache for all of them. One patient has taken aspirin for prevention, and recurrent 3 years later; two patients did not take medicine, and recurrent 2 and 3 years later, separately; and 2 patients taken warfarin, and recurrent 2 and 8 years later, separately. Come to these conclusions, we considered that the recurrent rate may relate to the follow-up period, which may not be long enough; or may be due to insufficient sample size, further studies are needed, and subgroup analysis is necessary, to maximum benefit.

There are several limitations in our study. First, it is a retrospective study, not a randomized trial and, thus, more susceptible to bias. Second, some patients were evaluated only by phone at follow-up. Finally, the sample size was relatively small and potentially underpowered to assess for differences beyond that of the outcome for independence.

## 5. Conclusions

Our study reinforces the finding that outcomes after CVST are generally good, with the majority of patients achieving functional independence and a lower risk of recurrent events. For the patients over 40-year-old, motor or sensory deficit and altered consciousness were more common, and the hemorrhage rate and mortality rate were higher than the younger patients. A further dedicated study is needed.

## Figures and Tables

**Figure 1:** Modified Rankin Scale distribution by selected patient groups.

**Figure 2:** Schematic diagram of cerebral venous sinus thrombosis locations and distribution.

**Table 1:** Baseline characteristics of CVST patients.

	Total (113)	Age < 40 (65)	Age ≥ 40 (48)	*p*
Median age = 32.50 (IQR 27-48.75)				
Female, *n* (%)	63 (55.75%)	41 (63.07%)	22 (44.83%)	0.600
Follow-up period	10 m (6-24 months)			
Medical encounter lag time^∗^	0.04 d-120 d (average11.11)	12.48	9.26	
Median time (IQR)	5.00 (2.00-10.00)	4.50 (2.25-9.75)	5.00 (2.00-14.00)	<0.01
Symptoms and signs, *n* (%)				
Headache	98 (86.72%)	61 (93.84%)	37 (77.08%)	0.01
Visual loss	10 (8.85%)	8 (12.31%)	2 (4.17%)	0.18
Papilledema	17 (15.04%)	12 (18.46%)	5 (10.42%)	0.29
Nausea/vomiting	64 (56.63%)	39 (60.00%)	25 (52.08%)	0.44
Stupor or coma	12 (10.62%)	4 (6.15%)	8 (16.67%)	0.12
Motor or sensory deficit	25 (22.12%)	13 (20.00%)	12 (25.00%)	0.64
Seizure	20 (17.70%)	13 (20.00%)	7 (14.6%)	0.61
NIHSS score > 2	28 (24.78%)	16 (24.61%)	12 (25.0%)	1.00
Risk factors				
None identified	36 (31.86%)	7 (10.77%)	29 (60.42%)	<0.01
Malignancy	3 (2.65%)	2 (3.07%)	1 (2.08%)	1.00
Dural fistula	1 (0.88%)	0 (0.00%)	1 (2.08%)	0.42
Coagulation disorder	14 (12.39%)	8 (12.31%)	6 (12.50%)	1.00
Any systemic prothrombotic disorder	8 (7.08%)	6 (9.23%)	2 (4.17%)	0.46
Polycythemia	2 (1.77%)	1 (1.53%)	1 (2.08%)	1.00
Anemia	8 (7.08%)	8 (12.31%)	0 (0.00%)	0.02
Pregnancy/puerperium	22 (19.47%)	22 (33.84%)	0 (0.00%)	<0.01
Local infection	31 (27.43%)	19 (29.23%)	12 (25.00%)	0.67
Oral contraceptives	3 (2.65%)	3 (4.61%)	0 (0.00%)	0.26
Surgery	8 (7.08%)	8 (12.31%)	0 (0.00%)	0.02
Dehydration	1 (0.88%)	1 (1.53%)	0 (0.0%)	1.00
mRS < 2	94 (83.18%)	55 (84.61%)	39 (81.25%)	0.80
Death by 6 month	3 (2.65%)	1 (1.53%)	2 (4.16%)	0.57
CVST recurrent	10 (8.85%)	4 (6.15%)	6 (12.50%)	0.31

^∗^Medical encounter lag time (from symptom onset to first medical encounter).

**Table 2:** Imaging findings of CVST patients.

	Total (113)	Age < 40 (65)	Age > 40 (48)	*p*
Neuroimaging at admission				
CT/MRI showed infarct, *n* (%)	21 (18.58%)	10 (15.38%)	11 (22.92%)	0.33
CT/MRI showed hemorrhage, *n* (%)	17 (15.04%)	7 (10.77%)	10 (20.83%)	0.18
Occluded sinus/vein, *n* (%)				
Superior sagittal sinus	60 (53.10%)	31 (47.69%)	29 (60.42%)	0.18
Straight sinus	8 (7.08%)	3 (4.61%)	5 (10.42%)	0.28
Sigmoid sinus	57 (50.44%)	34 (52.31%)	23 (47.92%)	0.70
Transverse sinuses	55 (48.67%)	31 (47.69%)	24 (50.00%)	0.85
Number of affect sinus, *n* (%)				
One sinus	47 (41.59%)	26 (40.00%)	21 (43.75%)	0.70
Two sinuses	40 (35.40%)	24 (36.92%)	16 (33.33%)	0.84
More than two sinuses	26 (23.00%)	12 (18.46%)	14 (29.17%)	0.25

## Data Availability

The data used to support the findings of this study are available from the corresponding author upon request.
